This article has been retracted.

# CNN-GRU-AM for Shared Bicycles Demand Forecasting

**DOI:** 10.1155/2021/5486328

**Published:** 2021-12-06

**Authors:** Yali Peng, Ting Liang, Xiaojiang Hao, Yu Chen, Shicheng Li, Yugen Yi

**Affiliations:** School of Software, Jiangxi Normal University, Nanchang 330022, China

## Abstract

The demand forecast of shared bicycles directly determines the utilization rate of vehicles and projects operation benefits. Accurate prediction based on the existing operating data can reduce unnecessary delivery. Since the use of shared bicycles is susceptible to time dependence and external factors, most of the existing works only consider some of the attributes of shared bicycles, resulting in insufficient modeling and unsatisfactory prediction performance. In order to address the aforementioned limitations, this paper establishes a novelty prediction model based on convolutional recurrent neural network with the attention mechanism named as CNN-GRU-AM. There are four parts in the proposed CNN-GRU-AM model. First, a convolutional neural network (CNN) with two layers is used to extract local features from the multiple sources data. Second, the gated recurrent unit (GRU) is employed to capture the time-series relationships of the output data of CNN. Third, the attention mechanism (AM) is introduced to mining the potential relationships of the series features, in which different weights will be assigned to the corresponding features according to their importance. At last, a fully connected layer with three layers is added to learn features and output the prediction results. To evaluate the performance of the proposed method, we conducted massive experiments on two datasets including a real mobile bicycle data and a public shared bicycle data. The experimental results show that the prediction performance of the proposed model is better than other prediction models, indicating the significance of the social benefits.

## 1. Introduction

With the continuous acceleration of urbanization and the expansion of the scale of cities, the pressure on transportation is increasing. In order to reduce the pressure on road traffic and solve the increasingly serious traffic problems, various localities have proposed the travel mode of “rail + bus + slow travel.” Public bicycles have been developed due to their own characteristics including green, pollution-free, low energy consumption, and small footprint, which have been vigorously promoted by governments in recent years [1]. As an extension of public bicycles, shared bicycles have been widely used and developed in many cities all over the world [2]. However, with the rapid development of shared bicycles, fluctuations in temporal and spatial demand have led to an uneven distribution of urban vehicles, such as “oversupply” in some areas and “supply exceeds demand” in other areas [3].

To address the aforementioned problems, it is necessary to predict the demand for each operating area of shared bicycles and arrange the vehicle scheduling among the areas reasonably. At present, a lot of research studies on the accuracy of bicycle demand forecasting have been carried out. They can be divided into two classes: one is the users' choice of the travel model and another is the key influence factors. In the study of the users' travel options, Campbell et al. [4] investigated the users' travel mode and smart card data to identify the important factors that affect the users' travel frequency. El-Assi et al. [5] used a distributed lag model to evaluate the impact of the built environment and weather on the demand for shared bicycles in Toronto. This model links the number of daily public bicycle trips at the site with land utilization, built environment, and weather conditions. Fournier et al. [6] used a sine model to predict seasonal shared bicycle demand. For another, in the study of key influencing factors [7], Eren and Uz [8] proposed a framework for comprehensively displaying the influencing factors of shared bicycle travel demand, which was used to evaluate the impact of various factors on the demand for car borrowing at the site. The experimental results demonstrated that weather and geographic location factors play a key role in the prediction results. Gebhart and Noland [9] used hourly weather data to assess the impact of weather conditions on shared bicycle travel patterns. Cold weather and high humidity will reduce the demand for bicycle rental. The above results provide valuable insights for analyzing the key factors affecting the demand for shared bicycles.

Recently, deep learning is widely used in time-series forecasting [10–16]. The bicycle-sharing demand forecasting is a forecasting problem of spatiotemporal data which contains spatial and temporal attributes. For the spatial attributes, Kang et al. [10] fully considered the spatial complexity, nonlinearity, and uncertainty of the transportation network and proposed a convolutional neural network prediction model. This model effectively uses the spatial information of the traffic data, but it ignores the time attributes. Therefore, Zhang et al. [11] comprehensively considered time and space information and proposed a prediction model based on convolution and residual networks, which makes the prediction results more accurate. For the temporal attributes, Fu et al. [12] used long short-term memory (LSTM) and its variant network gated recurrent unit (GRU) to predict short-term traffic flow. Furthermore, Yu et al. [13] applied LSTM and autoencoder to capture the time dependence of traffic prediction under extreme conditions and proposed a traffic flow LSTM neural network forecast model. Xu et al. [14] used big data analysis and LSTM model to predict the demands for shared bicycles. The above studies have analyzed the demand for shared bicycles from the perspectives of time and space. Both CNN and LSTM have advantages in extracting feature information, but they have the disadvantage of weak interpretability. In recent years, the attention mechanism has been widely used in various fields of deep learning. Combining the attention mechanism, the accuracy and training speed of the deep learning model have been greatly improved. For example, Bahdanau et al. [15] introduced an attention mechanism in the process of acquiring semantic features, which improved the accuracy of translation. Xu et al. [16] established two attention mechanisms, namely, “soft” and “hard,” and explained the process of generating model weights. The above studies have shown that the attention mechanism has a huge effect on sequence learning tasks. Therefore, attention mechanism is applied to the demand forecast of shared bicycles, where the different weights are assigned to different factors and can help to reduce the error value and improve the performance of the bicycle demand forecasting model.

In summary, to overcome the problems of incomplete consideration and insufficient forecasting algorithms in traditional bicycle demand forecasting, that is, only considered one aspect of time or space attributes [17, 18], this paper proposes a shared bicycle demand prediction model based on convolutional recurrent neural network with the attention mechanism named as CNN-GRU-AM. We not only consider the volatility of historical travel data of users but also analyze the impact of users' travel characteristics and external factors on the demand for shared bicycles.

The rest of paper is organized as follows. In Section 2, the data processing and influencing factors' analysis are introduced. The proposed method is introduced in Section 3. In Section 4, extensive experiments on two datasets are conducted to evaluate the performance of the proposed method. Finally, the conclusions and further works of our study are described in Section 5.

## 2. Data Processing and Influencing Factors' Analysis

### 2.1. Operating Area and Data Processing

Shenzhen is located on the southern coast of China, with geographic coordinates between 113°46′ to 114°37′ east longitude and 22°27′ to 22°52′ north latitude. According to the geographic location information of the operation area, the shaded part in Figure 1 can be divided into five parts. Among them, A is Nanshan District, which includes four operating areas such as Nanshan, Shekou Street, Yuehai Street, and Merchants Street. B is Longhua District, which includes three operating areas of Dalang Office, Guanlan Office, and Longhua Office. C is Futian District which only has Fubao Street operating area. D is Longgang District, which contains Henggang Street, Longgang Central City, and Minzhi Office operating areas. E is Pingshan District, which includes Pingshan Street and Kengzi Street operating areas.

Shared bicycles can only be rented and returned by scanning the code through the APP in any operating area. As of December 2018, Shenzhen has launched 6,720 shared bicycles which are used approximately 4,353.33 times per day, bringing the significant social and environmental benefits. Combined with wave-front theory, we have proposed an accessibility index capacity potential evaluation model to select key nodes [19]. The key node is that users' demand is large, and the problem nodes of “supply exceeds demand,” and “oversupply” often occurs in the morning and evening peaks. The dataset is the real data of three operating areas in Shenzhen from July 2016 to July 2017, which are obtained by the hardware equipment uploaded to the city's bicycle-sharing system. However, the system sometimes encounters problems with equipment such as power failure and network disconnection, resulting in some data loss. At the same time, due to manual scheduling and user inspections before daily use, a lot of invalid data will be generated. They mainly include the following. (1) The borrowing time is less than or equal to 1 minute, which can be inferred as vehicle inspection data. (2) Data with a bicycle duration longer than 24 hours can be considered as abnormal borrowing data such as bicycle stolen and repaired. (3) Most of the bicycle users are sleeping at 0 am–5 am, and the number of borrowed bicycles generated is small, so this data of the time period has little influence on the model prediction results. Therefore, the above unreasonable data needs to be eliminated. The results of data preprocessing are shown in Table 1.

### 2.2. Analysis of Influencing Factors

#### 2.2.1. Analysis of Temporal and Spatial Characteristics

From the time dimension, we can find out that the usage of shared bicycles in various time periods determines whether there will be a shortage within a short period of time. As shown in Figure 2, the demand for bicycles has cyclical changes on working days and rest days. It is obvious that morning and evening are peaking on working days, and the number of vehicles used during the peak period increases sharply, while the rest days are flat relatively and no obvious peak period.

From the spatial dimension, the hotspots of shared bicycles are mainly concentrated on high-density and high-intensity travel activities during workdays. At the same time, along the metro or bus station, the residential quarters, and the business districts are high-frequency cycling areas for shared bicycles, which show that city-sharing bicycles mainly solve the problem of urban “last mile” travel.

#### 2.2.2. Analysis of Weather Characteristic Factors

In addition to the aforementioned factors, weather conditions also have a greater impact on the demand of shared bicycles [20].  Table 2 shows the weather components in the study. The data come from the National Meteorological Center.

The Pearson correlation coefficient that measures the correlation between two variables is a numerical value [21]. Its range is from −1 to 1, where 1 means complete agreement and −1 means complete inconsistency. The larger the coefficient value, the stronger the correlation. The calculation method is that the covariance of two variables is divided by the standard deviation of the two variables, and the calculation formula is as follows:

(1) $$\begin{array}{c} \rho_{X,Y}=\frac{E\left(XY\right)-E\left(X\right)E\left(Y\right)}{\sqrt{E\left(X^{2}\right)-E^{2}\left(X\right)}-\sqrt{E\left(Y^{2}\right)-E^{2}\left(Y\right)}}. \end{array}$$

Sorting out the weather data and the historical travel data of shared bicycles, the Pearson correlation analysis between the number of borrowed bicycles and the above indicators was carried out, and the results are shown in Table 3.

From Table 3, the number of shared bicycle borrowings is strongly correlated with the number of users and is significantly correlated with other factors, indicating that the user's bicycle demand has a great correlation with weather conditions. Therefore, taking the time characteristics and weather conditions into account, it will be improve the accuracy of the demand forecast of shared bicycles.

## 3. The Proposed Method

Generally, the state of public transportation has a strong time dependence [22]. Shared bicycles can be regarded as one of the public transportations, so the demand of bicycle borrowing is also existing time dependent. Under normal circumstances, the time dependent trend will follow a certain historical pattern. In the same pattern, weather conditions also have a great impact on the demand for shared bicycles. Therefore, in order to improve the prediction accuracy and vehicle scheduling efficiency, this paper proposes a CNN-GRU-AM network prediction model. The overall frame diagram is shown in Figure 3.

As shown in Figure 3, the input data consist of three parts, including historical travel data of shared bicycles, time characteristic data and weather data. This model mainly consists of four parts. Firstly, the input data that are sent to the two-layer CNN network to extract the features. Secondly, the outputs of CNNs network are regarded as the input data of the GRU network, which can be trained by a large amount of data to find the proper parameters. Therefore, GRU can learn the time-series relationship among these features. Thirdly, the attention mechanism is introduced to get the degree of importance of the above features, which can obtain the weighted features in the network. Finally, a fully connected network with three layers is used to obtain the forecast results of shared bicycle demand.

### 3.1. CNN Network

Convolutional neural networks (CNN) [23] have strong feature extraction capabilities, which can extract the relationship between multidimensional time-series data in the spatial structure. In CNN, local key information can be extracted effectively by setting different convolution kernels. Then, the usage of local connections and weight sharing can reduce the number of the training parameters and the complexity of the model, so as to improve the model efficiency [24]. The typical convolutional neural network structure is shown in Figure 4.

CNN has made great research results in the processing of two-dimensional images; it can also be widely used to process one-dimensional data [25]. In our proposed method, we only use the convolutional layer to extract the features from the data. In the convolutional layer, the input data need to perform the convolution and activation operations. The calculation formula is as follows:

(2) $$\begin{array}{c} X_{t}=\sigma \left(Wx_{t}+b\right), \end{array}$$

where *W* is the weight coefficient of the filter, *x*_*t*_ is the *t*th input data, and *X*_*t*_ is the output result of *x*_*t*_.

### 3.2. GRU Network

For a period of time in the future, the bicycle demand of the user will be affected by the current and previous status of the bicycle. Therefore, in order to remember the bicycle status of a long time ago, this paper studies the influence of different time steps on the demand of the next bicycle. Long short-term memory (LSTM) [26] is based on the recurrent neural network (RNN) [27] architecture, which aims to solve the problem of long-term dependence of RNN. It can be better captured the complex nonlinear relationship in time-series data [28]. Gated recurrent unit (GRU) [29] is a variant of LSTM which composes of an update gate *z*_*t*_ and a reset gate *r*_*t*_. The update gate is used to determine the information to be discarded and the new information needs to be added. The reset gate determines the degree of the previous information which is discarded. The network structures of LSTM and GRU are shown in Figure 5.

Compared with LSTM, GRU has a simple structure and utilizes two gated switches to achieve better performance than LSTM. Since the number of gate is less than that of LSTM, the number of parameters is reduced, so the risk of overfitting is reduced. Theerawit et al. [30] applied CNN-GRU and CNN-LSTM to emotion recognition and found that the performance of them is similar, but the training time of CNN-GRU is faster. Therefore, this paper chooses GRU for modeling.

Take the output of the CNN layer *X* = {*x*_1_, *x*_2_,…, *x*_*t*_} as the input of the GRU time series. *H* = {*h*_1_, *h*_2_,…, *h*_*t*_} is the output of the hidden layer, which is the demand forecast result. The hidden layer unit *h*_*t*_ of GRU can be calculated by the following formula:

(3) $$\begin{array}{c} z_{t}=\sigma \left(W_{z}x_{t}+U_{z}h_{t-1}\right),\\ r_{t}=\sigma \left(W_{r}x_{t}+U_{r}h_{t-1}\right),\\ {\tilde{h}}_{t}=\tanh\left(r_{t}*U_{r}h_{t-1}+Wx_{t}\right),\\ h_{t}=\left(1-z_{t}\right)*{\tilde{h}}_{t}+z_{t}*h_{t-1}, \end{array}$$

where *W*_*z*_ and *W*_*r*_ and *U*_*z*_ and *U*_*r*_ represent the weight matrix of *x*_*t*_ and *h*_*t*−1_, respectively, *W* is the training parameter matrix, *x*_*t*_ is the time-series data of the current time interval *t*, *h*_*t*−1_ is the output of the memory unit in the previous time interval *t* – 1, *σ* is the sigmoid function, and tanh is the hyperbolic tangent function. The calculation formula is as follows:

(4) $$\begin{array}{c} \text{sigmoid}=\frac{1}{1+e^{-x}},\\ \tanh=\frac{e^{x}-e^{-x}}{e^{x}+e^{-x}}. \end{array}$$

In this paper, we add a layer of GRU with 64 hidden neurons behind the two layers of CNN. The activation function is sigmoid, which is used to learn the time-series relationship between data. Thus, effective dynamic modeling can be performed on the time-series data of shared bicycles.

### 3.3. Attention Mechanism

Attention mechanism (AM) [31, 32] is derived from the study of human vision, and it mainly includes two aspects: (1) deciding to focus on the input part and (2) allocating limited resources to important parts. In recent years, the attention mechanism has been widely used in the modeling of prediction tasks, which can assign different weights to the hidden layers according to the influence of different features on the output. In order to pay attention to the impact of different input characteristics on the prediction results, the attention mechanism is introduced into the shared bicycle demand prediction model to improve the prediction accuracy in this paper. AM keeps the intermediate output results of the previous network layer firstly and then associates them with the value of the output sequence. In this way, this model is trained to select the input features that need to be focused, which gives higher weight to the input features with high relevance.  Figure 6 is a schematic diagram of the attention mechanism.

The weight calculation formula is as follows:

(5) $$\begin{array}{c} u_{t}=\tanh\left(w_{i}h_{t}+b\right),\\ a_{t}=\text{softmax}\left(u_{t}^{T},u_{w}\right), \end{array}$$

where *w*_*i*_ is the weight matrix, *h*_*t*_ is the output vector of the hidden layer of the GRU, *u*_*t*_ is the activation vector of *h*_*t*_, and *a*_*t*_ is the assigned weight value.

Once *a*_*t*_ and *h*_*t*_ are obtained, the final vector *A*_*t*_ can be obtained as follows:

(6) $$\begin{array}{c} A_{n}=\sum_{t=1}^{T}a_{t}u_{t}. \end{array}$$

## 4. Experimental Analysis

This experiment is performed on PC machine with Intel(R) Core(TM) i5-8265U CPU@1.60 GHz 1.80 GHz and 16 GB memory and Windows 10 operating system. The programming language is Python with the version number is 3.7.4. The integrated development environment (IDE) is PyCharm, and machine learning libraries including Tensorflow (2.1.0) and Keras (2.3.1) are used to implement all the algorithms.

### 4.1. Datasets

A real shared bicycle dataset in three operating areas in Shenzhen and a public shared bicycle dataset in Washington are employed in this experiment. Each dataset includes shared bicycle historical travel data, time characteristic data, and weather data. Tables 4 and 5 show the description and feature description of the datasets, respectively.

The preprocess of the data is needed to be preformed. In this work, the one-hot encoding is utilized to encode working and hour characteristics. The historical travel data of shared bicycles and weather data are normalized to [0, 1] through the minimum and maximum normalization method. The conversion formula is as follows:

(7) $$\begin{array}{c} X=\frac{x-x_{\min}}{x_{\max}-x_{\min}}, \end{array}$$

where *x* is the original feature, *X* is the normalized vector of *x*, and *x*_min_ and *x*_max_ are the minimum value and the maximum value of the current vector *x*, respectively.

### 4.2. Model Evaluation Indicators

In order to quantitatively analyze the accuracy and superiority of the model, the root mean square error (RMSE), mean absolute error (MAE), and average percentage error (MAPE) [33] are employed to measure the performance of different evaluation indicators on different prediction models. More specifically, RMSE and MAE measure the absolute magnitude of the deviation between the true value and the predicted value, and MAPE measures the relative magnitude of the deviation. In addition, MAE and MAPE are not easily affected by extreme values. RMSE is computed by the square of the error, but it is more sensitive to outlier data. Most of methods adopted these indicators due to their own advantages. Thence, the above indicators are to measure the difference between the predicted value and the true value of the number of shared bicycles. The calculation formula is as follows:

(8) $$\begin{array}{c} \text{RMSE}=\sqrt{\frac{1}{n}\sum_{i=1}^{n}{\left(y_{i}-{\hat{y}}_{i}\right)}^{2}},\\ \text{MAE}=\frac{1}{n}\sum_{i=1}^{n}\left|y_{i}-{\hat{y}}_{i}\right|,\\ \text{MAPE}=\frac{1}{n}\sum_{i=1}^{n}\frac{\left|y_{i}-{\hat{y}}_{i}\right|}{{\hat{y}}_{i}}, \end{array}$$

where *y*_*i*_ and ${\hat{y}}_{i}$ are the actual value and the predicted value, respectively, and *n* is the number of samples. In the forecast of the demand for shared bicycles, the smaller the RMSE, MAE, and MAPE values, the smaller the forecast error value and the more accurate the forecast result. In this paper, we mainly use the MAPE value to train the neural network and also refer to the changes of the other two values.

### 4.3. Model Training Parameter Settings

There are four parts in the proposed model, namely, CNN layer, GRU layer, AM layer, and fully connected (FC) layer. The activation function of the GRU layer in the model is sigmoid, and the activation functions of the other three layers are all ReLU. The optimizer chooses Adam, the learning rate is set to 0.0001, and the model is trained for 70 rounds (Epochs). The setting of the convolutional layer parameters will affect the performance of the model. We have conducted experiments on the number of layers of the convolutional layer, the size of the filter, and the value of the kernel parameters.  Table 6 shows that the number of convolutional layers is 1. When the size of filter and kernels are set as 128 and 1, the experimental results of the proposed method on the three datasets are the best.  Table 7 shows that the number of convolutional layers is 2. From this table, when the sizes of filter of two-layer CNN layer are set as 128 and 64, and the kernels_size is set to 1, the experimental results of the proposed method on the three datasets are optimal.

In our model, the other two main parameters, i.e., time_step and batch_size, are affected by the prediction performance.  Table 8 shows the average error values of the three datasets when time_step and batch_size take different values.

From Table 8, when the time_step is set to 10 and batch_size is set to 256, the experimental prediction error value is the smallest and the accuracy is the highest. Therefore, these values will be used in the subsequent model comparison experiment.

### 4.4. Experimental Results

#### 4.4.1. Experimental Results of a Real Shared Bicycle Dataset in Shenzhen

In order to verify the prediction performance of the proposed CNN-GRU-AM method, we compare it with the following prediction model.

1. LSTM [15]: LSTM considers the time series features in the dataset
2. GRU [33]: GRU is a variant of LSTM
3. CNN [34]: CNN considers the spatial information-weather feature in the dataset
4. GRU-CNN [35]: GRU-CNN is a hybrid model, in which GRU first is used to extract the time-series information of the input data, and then, CNN is applied to extract the weather features
5. CNN-GRU: CNN -CRU is a hybrid model, in which CNN is used to extract weather features, and then, GRU is applied to extract the time-series information

The prediction results of CNN-GRU-AM and the above compared prediction models on the three areas are shown in Table 9.

From Table 9, the CNN-GRU-AM model has the best performance on the three areas, which greatly improves the prediction performance of the model. LSTM is a deep learning network that can effectively obtain the temporal characteristics of long input sequences. However, it does not include a convolution unit, which cannot obtain spatial relationships. GRU is a variant of LSTM, which have better performance on some smaller data. Therefore, the prediction results of GRU are better than LSTM. Since the data have a strong correlation with the temporal characteristics, CNN can only extract local key information in space, and it also fails to take the temporal characteristics into account. Furthermore, comparing with the GRU-CNN model, the CNN-GRU model can be better prediction performance. The CNN-GRU model utilized CNN to extract local features in the data firstly and then uses GRU to extract time-series features for prediction, which can combine weather features with time-series features. More importantly, the proposed CNN-GRU-AM model introduces an attention mechanism into CNN-GRU, which assigns different weights to each feature by calculating the attention score. Therefore, it can identify the influential features that have a greater impact on the prediction results effectively and assign them bigger weight. Compared with the CNN-GRU model, the three prediction error values (RMSE, MAE, and MAPE) of the proposed model have been reduced in the three areas, especially the MAPE values have been decreased by 9.48%, 1.94%, and 2.22%, respectively. In summary, the prediction error values of the CNN-GRU-AM model are less than that of other prediction models, which improves the prediction accuracy. In order to show the performance more clearly, 300 data values randomly selected from the test results are shown in Figures 7–9. In this figure, the red curve is the real demand value of shared bicycles, and the blue curve is the predicted value. The horizontal axis is the selected test values at different time periods, and the vertical axis is the demand for the shared bicycle borrowing. From these figures, we can clearly see that the performances of the proposed CNN-GRU-AM outperform other compared method.

Then, the residual network (ResNet) can improve the accuracy by increasing a certain depth. The internal residual block of ResNet can effectively alleviate the problem of gradient disappearance caused by increasing depth in the deep neural network. We replaced the convolutional network with a residual neural network in the model. The experimental results are shown in Table 10. From this table, we found that the error value has changed significantly, but the overall forecast error value has not changed too much. In this paper, the number of data and model layers is small, so the prediction error value is smaller, and the prediction result is more accurate. Comparing with Table 9, the performance of the CNN-GRU-AM model is better than those of the ResNet-GRU-AM model.

#### 4.4.2. Experimental Results of the Public Bicycle Dataset in Washington

Since our datasets have not been made public, there is no relevant literature citing our dataset for research currently. In order to verify the prediction performance of the proposed CNN-GRU-AM model in this paper, the public shared bicycle dataset in Washington is introduced, which is a classic public dataset in the field of public bicycles. A large number of researchers have studied the demand forecast of this bicycle dataset already. We compare the previous research results with our method, and the characteristics of the dataset selected in the experiment are consistent with the three areas. The experiment is compared with the classic traffic flow prediction method:

1. HA [36]: the historical average method is a classic time prediction method. In the same time interval, it uses the average value of historical inflows and outflows to make predictions.
2. ARIMA [37]: ARIMA is a popular time-series forecasting model. It is simple and does not require other exogenous variables.
3. LSTM: LSTM is often used in time-series forecasting problems, which can capture long-term time dependent problems.
4. ASTRCNs [38]: The full name is the spatiotemporal loop convolutional network model based on the attention mechanism. Combined with the attention mechanism, it can adjust the importance of historical data to the prediction target dynamically.

The experimental results of the above prediction method on the Washington dataset are shown in Table 11.

The experimental results of the above methods on the three datasets in Shenzhen are shown in Table 12.

It can be obtained from the above tables, the experimental results of the proposed model are better than the classic time-series prediction model, so the CNN-GRU-AM model proposed in this paper can reduce the prediction error value and improve the predictive performance.

## 5. Conclusion

This paper takes Shenzhen shared bicycles as the research object and proposes a convolutional recurrent neural network prediction model based on the attention mechanism. In this model, CNN is used to learn and extract the local features. These features as the input of GRU are used to capture the time-series characteristics. Then, the attention mechanism is applied to extract the attention score of the output information of CNN-GRU, and the important feature factors are given greater weights. Finally, the output layer is integrated with three fully connected layers to predict the demand for shared bicycles. Experimental results show that the prediction performance of the proposed CNN-GRU-AM model on two datasets is also better than the comparison model. Furthermore, the effects of different experimental parameters on the model are also explored. The verified results show that the input features and attention mechanisms are effective to improve model performance, indicating the importance of time characteristics and external factors in predicting the demand for shared bicycles.

In the future work, we will explore other related factors (i.e., the population, the borrowing and repayment requirements of neighboring key stations, the public transportation connections around the stations, etc.) that affect the use of vehicles furtherly and continue to research more effective neural network methods. Furthermore, we will apply them to solve the time-series data and provide a theoretical basis for the scientific scheduling of time-series data.

## Figures and Tables

**Figure 1:** Distribution of public bicycle system outlets in Shenzhen.

**Figure 2:** The use of shared bicycles. (a) Working day. (b) Weekends or holidays.

**Figure 3:** The model structure of the proposed method.

**Figure 4:** The structure of typical CNN network.

**Figure 5:** The network structures of (a) LSTM and (b) GRU.

**Figure 6:** Schematic diagram of attention mechanism.

**Figure 7:** The prediction results of different models in Longgang Central City. (a) LSTM. (b) GRU. (c) CNN. (d) GRU-CNN. (e) CNN-GRU. (f) CNN-GRU-AM.

**Figure 8:** The prediction results of different models in Pingshang Street. (a) LSTM. (b) GRU. (c) CNN. (d) GRU-CNN. (e) CNN-GRU. (f) CNN-GRU-AM.

**Figure 9:** The prediction results of different models in Zhaoshang Street. (a) LSTM. (b) GRU. (c) CNN. (d) GRU-CNN. (e) CNN-GRU. (f) CNN-GRU-AM.

**Table 1:** Operational data elimination.

Data introduction	Longgang Central City	Pingshan Street	Zhaoshang Street
Total operating data	439092	617417	24922
Lending time ≤ 1 minute	1742	394	545
Lending time > 1440 minutes	1347	393	702
0 am–5 am	2104	3598	1376
Effective operation data	433899	613032	246599

**Table 2:** Descriptions of the weather components.

Influencing factors	Average value	Max	Min
Temperature (°C/day)	23	36.9	8.3
Precipitation (mm/day)	1935.8	3270	0
Wind speed (1 m/s)	5	12.1	1
Humidity (1%)	74	—	15

**Table 3:** Correlation between vehicle usage and weather conditions.

Correlation	Number of users	Number of borrowed bicycles	Temperature	Precipitation	Wind speed	Humidity
Number of users	—	0.993	0.55	0.528	0.543	0.431
Number of borrowed bicycles	0.993	—	0.521	0.526	0.549	0.448

**Table 4:** The description of the datasets.

Data	Time	Quantity	Hourly processing
Longgang Central City	2016.6–2017.8 (except Dec.)	433899	6935
Pingshan Street	2016.7–2017.8 (except Dec.)	613032	6935
Zhaoshang Street	2016.7–2016.11	246599	2907
Bicycle sharing in Washington	2011.1–2012.12	17380	17380

**Table 5:** Characteristic description of the datasets.

Characteristics	Value range and description
Temperature	[8.3, 36.8] unit: °C
Precipitation	[0, 3270] unit: mm
Wind speed	[1, 12.1] unit: m/s
Humidity	[15, /] average: 74 unit: 1%
Working	1/2 {1: working day; 2: (b) weekends/holidays}
Hour	5∼23 {5: 5 o'clock; 6: 6 o'clock; …; 23: 23 o'clock}

**Table 6:** Experimental results with the number of convolutional layer is 1 on three datasets.

Filter_size	Kernel_size	Longgang Central City			Pingshan Street			Zhaoshang Street		
		RMSE	MAE	MAPE	RMSE	MAE	MAPE	RMSE	MAE	MAPE
64	1	27.97	18.82	103.61	15.78	11.72	15.89	34.85	23.84	43.86
64	2	34.66	23.67	136.83	16.51	12.37	17.21	33.31	22.67	53.87
**128**	**1**	**26.67**	**16.65**	**63.78**	**14.02**	**10.36**	**14.15**	**31.88**	**21.68**	**39.60**
128	2	34.14	21.45	80.31	15.48	11.50	16.25	32.48	21.83	44.91
256	1	27.54	18.46	80.54	16.08	11.93	16.20	32.27	22.31	47.79
256	2	28.22	19.29	105.93	16.14	12.22	18.69	32.91	22.71	62.02

**Table 7:** Experimental results with the number of convolutional layer is 2 on three datasets.

Number of layers	Filter_size	Longgang Central City			Pingshan Street			Zhaoshang Street		
		RMSE	MAE	MAPE	RMSE	MAE	MAPE	RMSE	MAE	MAPE
Level 1	128	**26.96**	**16.67**	**49.56**	**14.02**	**10.36**	**14.15**	**31.88**	**21.68**	**39.60**
Level 2	64									
Level 1	128	26.13	16.54	62.57	15.95	11.89	16.49	32.57	22.14	43.37
Level 2	128									
Level 1	128	26.53	17.26	81.02	15.75	11.96	17.67	31.13	21.18	55.88
Level 2	256									

**Table 8:** The average error values of the three datasets.

Time_step	Batch_size	Longgang Central City			Pingshan Street			Zhaoshang Street		
		RMSE	MAE	MAPE	RMSE	MAE	MAPE	RMSE	MAE	MAPE
5	128	26.98	17.08	82.25	16.21	12.25	18.26	34.87	24.37	48.24
	256	26.15	16.74	74.74	15.84	11.94	17.16	34.02	22.68	47.07
	512	27.24	17.84	87.93	16.32	12.19	17.84	35.82	24.36	59.33
**10**	128	27.09	17.18	76.57	15.62	11.47	15.88	33.70	22.74	47.81
	**256**	**25.99**	**16.39**	**53.93**	**15.02**	**11.06**	**15.10**	**33.04**	**22.47**	**42.39**
	512	25.83	16.41	67.87	15.45	11.27	15.15	32.47	22.74	44.53
15	128	28.38	19.51	104.67	17.42	13.32	19.03	37.11	25.07	71.74
	256	30.30	20.86	106.82	15.84	11.94	15.51	35.13	23.77	55.29
	512	30.75	21.44	108.85	16.70	12.49	22.16	38.03	25.70	78.12

**Table 9:** Performance comparison of different models on three datasets.

<!—Col Count:10>Models	Longgang Central City			Pingshan Street			Zhaoshang Street		
	RMSE	MAE	MAPE	RMSE	MAE	MAPE	RMSE	MAE	MAPE
LSTM	36.92	27.44	161.06	20.13	16.33	26.84	38.03	25.70	71.74
GRU	31.71	22.33	134.55	19.12	14.92	23.00	37.11	25.07	62.30
CNN	28.38	19.51	103.99	16.21	12.25	18.55	35.82	24.36	56.28
GRU-CNN	27.09	17.18	81.23	15.23	11.50	17.35	35.13	23.77	48.24
CNN-GRU	26.32	16.74	61.11	15.10	11.37	16.09	33.81	23.02	43.52
CNN-GRU-AM	**26.96**	**16.67**	**49.56**	**14.02**	**10.36**	**14.15**	**31.13**	**20.77**	**39.01**

**Table 10:** Experimental results of using ResNet.

Model	Longgang Central City			Pingshan Street			Zhaoshang Street		
	RMSE	MAE	MAPE	RMSE	MAE	MAPE	RMSE	MAE	MAPE
ResNet	30.38	21.12	105.86	17.29	13.28	20.85	35.25	24.02	57.24
GRU-ResNet	27.31	18.48	92.36	16.06	12.05	18.06	33.37	22.85	53.33
ResNet-GRU	29.39	18.44	73.36	15.66	11.67	16.4	34.55	24.15	47.47
ResNet-GRU-AM	**26.87**	**16.99**	**58.62**	**14.26**	**10.56**	**14.56**	**33.02**	**22.16**	**41.92**

**Table 11:** Experiment results of the different models on the public bicycle dataset.

Model	RMSE	MAE	MAPE
HA	66.31	44.55	42.81
ARIMA	62.62	42.3	30.85
LSTM	61.26	40.31	31.06
ASTRCNs	56.87	37.69	28.89
CNN-GRU-AM	**55.26**	**36.76**	**27.58**

**Table 12:** Experimental results of three datasets on the benchmark model.

Model	Longgang Central City			Pingshan Street			Zhaoshang Street		
	RMSE	MAE	MAPE	RMSE	MAE	MAPE	RMSE	MAE	MAPE
HA	40.01	29.09	171.14	20.94	16.99	28.27	43.78	29.75	77.79
ARIAM	32.16	23.06	136.63	17.59	13.82	23.03	34.99	23.89	62.33
LSTM	36.92	27.44	161.06	20.13	16.33	26.84	38.03	25.70	71.74
ASTRCNs	26.26	16.61	69.74	16.01	11.87	16.67	34.11	23.19	41.44
CNN-GRU-AM	**26.96**	**16.67**	**49.56**	**14.02**	**10.36**	**14.15**	**31.13**	**20.77**	**39.01**

## Data Availability

The network code and data are available from the corresponding author upon request.
